RETRACTED

# MHF1–2/CENP-S-X performs distinct roles in centromere metabolism and genetic recombination

**DOI:** 10.1098/rsob.130102

**Published:** 2013-09

**Authors:** Sonali Bhattacharjee, Fekret Osman, Laura Feeney, Alexander Lorenz, Claire Bryer, Matthew C. Whitby

**Affiliations:** Department of Biochemistry, University of Oxford, South Parks Road, Oxford OX1 3QU, UK

**Keywords:** anaphase bridge, centromere, DNA helicase, DNA replication, homologous recombination

## Abstract

The histone-fold proteins Mhf1/CENP-S and Mhf2/CENP-X perform two important functions in vertebrate cells. First, they are components of the constitutive centromere-associated network, aiding kinetochore assembly and function. Second, they work with the FANCM DNA translocase to promote DNA repair. However, it has been unclear whether there is crosstalk between these roles. We show that Mhf1 and Mhf2 in fission yeast, as in vertebrates, serve a dual function, aiding DNA repair/recombination and localizing to centromeres to promote chromosome segregation. Importantly, these functions are distinct, with the former being dependent on their interaction with the FANCM orthologue Fml1 and the latter not. Together with Fml1, they play a second role in aiding chromosome segregation by processing sister chromatid junctions. However, a failure of this activity does not manifest dramatically increased levels of chromosome missegregation due to the Mus81–Eme1 endonuclease, which acts as a failsafe to resolve DNA junctions before the end of mitosis.

## 2. Introduction

Homologous recombination (HR) is a fundamental process in chromosome biology, being deployed in various ways to facilitate the repair and tolerance of DNA lesions in which genetic information is lost or corrupted in both strands of the double helix (e.g. a DNA double-strand break; DSB). It also promotes genome duplication by enabling the restart of collapsed replication forks, and in most studied eukaryotes serves a crucial role during meiosis in establishing chiasmata that guide correct disjunction of the homologous chromosomes during the first meiotic division. A potential consequence of its action is the rearrangement of genetic material, which in the germline can have the desirable effect of driving genetic diversity, but in somatic cells can lead to the loss or alteration of gene function, which in turn can result in disease and death.

Many proteins contribute to the correct functioning of HR; however, among these are a core cohort that is directly responsible for catalysing the key DNA transactions that occur [1]. Included here are nucleases and DNA helicases that often work hand in hand to generate a region of single-stranded DNA (ssDNA) with an exposed 3′-OH terminus onto which the central recombinase Rad51 can load supported by various mediator and accessory proteins. Once bound, Rad51 catalyses invasion of its DNA into an intact homologous duplex, forming a displacement (D) loop where the 3′ end of the invading strand can be used to prime DNA synthesis. The end stages of HR involve either the dissociation or cleavage of the D-loop or its maturation into one or two Holliday junctions (HJs) that similarly can be processed by a variety of DNA helicases/translocases and structure-specific nucleases to disengage the recombining DNA molecules, enabling them to segregate during mitosis/meiosis.

RETRACTED

One of the core components of the HR machinery is the FANCM DNA translocase [2–4]. In humans, FANCM is encoded by one of 15 genes in which mutations can cause the rare genetic disease Fanconi anaemia (FA), characterized by progressive bone marrow failure, developmental problems and cancer proneness. At a cellular level, deficiencies in FA proteins result in hypersentivity to DNA interstrand cross-linking (ICL) agents such as cisplatin, increased chromosomal abnormalities, increased DNA bridges during mitosis, and high rates of bi- and multinucleated cells that result from failed cytokinesis [5]. The products of the FA genes are part of a DNA repair network with eight members (FANCA, -B, -C, -E, -F, -G, -L and -M), forming the so-called FA core complex that monoubiquitinates FANCD2 and FANCI, which in turn are thought to direct subsequent repair events involving HR and translesion DNA synthesis [6]. FANCM's role here is to target the core complex to sites of stalled replication, which promotes the monoubiquitination reaction [2,7–9]. However, various lines of evidence also point to key roles for FANCM in HR that are independent of core complex activation and FANCD2/I monoubiquitination [4]. Not least among these are studies of the yeast orthologues of FANCM (Mph1 in *Saccharomyces cerevisiae* and Fml1 in *Schizosaccharomyces pombe*), which operate in environments that are devoid of most other FA proteins.

FANCM, Mph1 and Fml1 are superfamily 2 DNA helicases/translocases, and *in vitro* can use the energy from hydrolysing ATP to drive fork remodelling, HJ branch migration and D-loop dissociation [10–15]. Based on the findings of cell biological and genetic experiments, it is thought that these activities are used to support at least two reactions related to HR *in vivo*, namely the reversal of stalled replication forks (which could be used to generate a substrate for HR to promote replication restart) and the processing of recombination intermediates that enables the recombining DNAs to disjoin. In the latter case, several studies have shown that FANCM and its orthologues can limit the formation of crossover (CO) recombinants that stem from the cleavage of D-loops/HJs by structure-specific nucleases such as Mus81–Eme1 [12–14,16–20]. COs are reciprocal exchanges of the chromosomal regions that flank the site at which HR has acted. In meiotic cells, they are necessary for the establishment of chiasmata, but in somatic cells they can result in deleterious genome rearrangements if the recombining DNAs are other than perfectly aligned sister chromatids. The ability of FANCM/Mph1/Fml1 to direct CO avoidance most probably relates to its D-loop dissociation activity, which negates the need for junction resolution by a nuclease, and, in the context of a DSB, drives repair via a sub-pathway of HR called synthesis-dependent strand annealing that generates only non-crossover (NCO) recombinants.

RETRACTED

Recently, it was found that FANCM interacts with a complex of two small histone-fold proteins named MHF1 and MHF2 (i.e. FANC*M*-associated *H*istone-*F*old protein 1 and 2) [21,22]. The interaction occurs via a region just on the C-terminal side of FANCM's helicase domain, which docks onto a heterotetramer configuration of MHF1 and MHF2 that resembles the H3–H4 heterotetramer within histone octamers [23]. For brevity, we will refer to both the yeast and human form of this complex as MHF henceforth. Genetic studies in HeLa and/or chicken DT40 cells have shown that MHF functions alongside FANCM in promoting FANCD2 monoubiquitination following induction of ICLs, and suppressing spontaneous sister chromatid exchange (SCE), albeit in the latter case not to the same extent as FANCM [21,22]. At least in part, it appears to fulfil these roles by promoting the stability, chromatin association and substrate targeting of FANCM. *In vitro* purified MHF binds to double-stranded DNA (dsDNA) and enhances the fork reversal activity of FANCM [21,22]. Intriguingly, there is a synergistic increase in the DNA binding activity of the FANCM–MHF complex, resulting from the establishment of an additional DNA binding site, which is presumably important for substrate targeting [22,23].

Interestingly, MHF1 and MHF2 are also components of the constitutive-centromere-associated network (CCAN), going under the names of CENP-S and CENP-X, respectively [24,25]. Here, they interact with CENP-T and CENP-W to form a stable heterotetramer that can wrap DNA around itself in a manner that is thought to be analogous to the tetrasome formed by the histone H3–H4 heterotetramer [25]. CENP-T interacts directly with the Ndc80 complex of the outer kinetochore, which in turn attaches to the microtubules of the mitotic spindle [26–28]. In this way, CENP-T-W-S-X is thought to form a point of anchorage for the kinetochore at the centromere that is additional to that formed by the interaction of Ndc80 to CENP-A-containing nucleosomes via Mis12 and CENP-C. DT40 cells deficient in MHF exhibit noticeable defects in kinetochore architecture, including reduced localization of Ndc80 to the outer kinetochore and an increase in the intrakinetochore distance between CENP-T and Ndc80, and depletion of MHF2 in HeLa cells results in numerous mitotic defects, including a high proportion of misaligned chromosomes at the metaphase plate [24].

RETRACTED

To gain a greater understanding of MHF's roles in DNA recombination and repair, and how this relates to its function at the centromere, we have conducted a genetic and biochemical analysis of *S. pombe* MHF. We show that MHF's DNA repair/recombination role is distinct from its centromeric role, with the former depending largely on its physical interaction with Fml1 and the latter being independent of Fml1. We also reveal that MHF is recruited to DNA bridges and trailing segments of DNA during mitosis in a Fml1-dependent manner. Impairment of Fml1's catalytic activity or interaction with MHF increases the frequency of mitotic DNA bridges, but relatively few of these lead to gross chromosome missegregation, seemingly due to processing by the Mus81–Eme1 endonuclease. Our data indicate that unresolved recombination intermediates often persist into mitosis and are processed by Fml1–MHF or Mus81–Eme1 even as late as anaphase/telophase.

## 3. Results

### 3.1. Mhf1 and Mhf2 localize to centromeres, and are needed for correct chromosome segregation during meiosis

In contrast to *fml1*, deletion of either *mhf1* or *mhf2* in fission yeast results in a marked reduction in growth and viability indicating that MHF performs a critical function that does not require Fml1 (figure 1*a*). Epifluorescence microscopy of strains expressing GFP-tagged forms of Mhf1 and Mhf2 show that they co-localize with the CCAN component Mis6 (CENP-I), confirming that Mhf1 and Mhf2 are centromeric proteins in fission yeast (figure 1*b*; electronic supplementary material, figure S1). Analysis of meiotic chromosome segregation using strains in which chromosome 2 is marked with an array of *lacO* sequences bound by the LacI repressor protein fused to GFP showed that deletion of *mhf2* results in a high proportion of meiosis I and II segregation defects (figure 1*c,d*). By contrast, a *fml1Δ* mutant exhibits almost wild-type levels of accuracy for meiotic chromosome segregation (figure 1*d*). Altogether these data are consistent with the notions that MHF plays an important role at the centromere in establishing proper kinetochore function, which is needed for faithful chromosome segregation, and that this function is independent of its involvement with Fml1 in recombination.

RETRACTED

**Figure 1.** MHF functions at the centromere and promotes viability and chromosome segregation independently of Fml1. (*a*) Spot assay showing the relative growth of strains MCW1221, MCW2080, MCW4639 and MCW4777 on YES agar after 3 days at 30°C. (*b*) Example cells from a culture of MCW5846 showing the co-localization of Mhf1-GFP with Mis6-mCherry. (*c*) Schematic of the meiotic chromosome segregation assay. (*d*) Meiotic chromosome segregation in asci from wild-type (AY167-1D × FO652), *fml1Δ* (MCW4172 × MCW6196) and *mhf2Δ* (MCW4777 × MCW5113) homozygous crosses.

### 3.2. MHF interacts with the C-terminal region of Fml1

Human MHF binds to a region on the C-terminal side of FANCM's helicase domain [22,23]. To see whether the same is true for the fission yeast orthologues, we established an *in vitro* assay for determining their interaction using purified MHF (figure 2; electronic supplementary material, figure S2A) and Fml1 fused to maltose binding protein (MBP). Essentially, MBP-Fml1 bound to amylose resin was tested for its ability to retain MHF on the resin, with detection of the complex on a Western blot using an antibody against a His-tag fused to Mhf2. As expected, full-length Fml1, which is 834 amino acids (figure 2*a*), retained MHF on the resin, whereas MBP or resin alone did not (figure 2*b*). We next tested various fragments of Fml1 for their ability to bind MHF; by this approach, we narrowed down the point of interaction to a region between amino acids, 620 and 700 (figure 2*a*,*b*; electronic supplementary material, figure S2B,C). Further division of this region established that amino acids 650–690 encompassed the site of interaction (figure 2*c*), and that amino acids 670–690 are sufficient to retain MHF on the resin, but only under conditions of limited washing (figure 2*d*). To identify key residues needed for the interaction, we chose to mutate the tyrosine and arginines in the 670–690 region to alanine as such changes have been shown to frequently disturb protein–protein interactions in other cases [29] (figure 2*e*). Three combinations of mutations were tested, and whereas changing arginines 683, 686 and 687 to alanine had no effect on the ability of the 650–690 amino acid fragment to interact with MHF, changing tyrosine 672 together with arginines 674 and 678 to alanine totally abolished binding both in the context of the 650–690 amino acid fragment and the full-length protein (figure 2*f*,*g*).

**Figure 2.** MHF interacts with Fml1. (*a*) Schematic of Fml1 and the various truncated forms of it used in (*b*) and (*c*). The position of the MBP fusion, DNA helicase motifs (blue bars), and region encompassing the site of MHF interaction (red box) are shown. The numbers refer to amino acid positions. (*b–d*) Western blots showing the amount of His-tagged Mhf2 retained on amylose resin that has been pre-incubated with the indicated MBP-Fml1 fragment (the numbers refer to amino acid positions). (*e*) Amino acids 670–690 in Fml1 with the mutations tested in (*f*) indicated. (*f*) Western blot showing the retention of His-tagged Mhf2 on amylose resin pre-incubated with MBP-Fml1^650–690^ or its mutant derivatives 1–3. (*g*) Western blot showing that full-length Fml1^AAA^ fused to MBP fails to retain HisMhf2 on amylose resin. (*h*) SDS-PAGE analysis of gel filtration fractions 32–38 from the purification of the Fml1^576–725^–MHF complex. The gel was stained with Coomassie blue. (*i*) EMSA comparing the ability of MHF and the Fml1^576–725^–MHF complex to bind linear dsDNA. The amounts of protein are 49 nM (lanes b and f), 98 nM (lanes c and g), 490 nM (lanes d and h) and 980 nM (lanes e and i).

RETRACTED

### 3.3. MHF's ability to bind dsDNA appears to be enhanced by its interaction with Fml1's C-terminal domain

It has recently been shown that the interaction between human MHF and FANCM generates a DNA binding site, which results in a synergistic increase in DNA binding of the protein complex [23]. To see whether the same is true for *S. pombe* MHF and Fml1, we co-expressed Fml1's C-terminal domain (residues 576–725) with Mhf1 and His-tagged Mhf2 in *Escherichia coli* and purified the complex by nickel affinity and gel filtration chromatography (figure 2*h*). We then compared the DNA binding ability of this complex to that of the MHF complex using an electrophoretic mobility shift assay (EMSA; figure 2*i*). The MHF complex without Fml1^576–725^ binds a 50 bp linear dsDNA to form a single retarded band at relatively high protein concentrations (greater than 1.48 µM; electronic supplementary material, figure S2D). By contrast, much lower concentrations of the MHF–Fml1^576–725^ complex (less than or equal to 490 nM) can achieve the same amount of DNA binding, consistent with the idea that the interaction between MHF and Fml1 forges an additional DNA binding site (figure 2*i*, lanes h and i). However, a caveat to this experiment is that we were unable to purify Fml1^576–725^ to homogeneity and therefore are uncertain whether or not this region of Fml1 binds DNA in its own right.

### 3.4. Fml1's ability to interact with MHF is important but not essential for its role in DNA repair

We have previously shown that Fml1 is needed for the repair/tolerance of DNA damage induced by the alkylating agent methyl methanesulfonate (MMS) and the DNA ICL agent cisplatin [12,14]. To see whether MHF also plays a role here alongside Fml1, we compared the MMS and cisplatin sensitivities of *fml1Δ*, *mhf1Δ* and *mhf2Δ* single and double mutant strains (figure 3*a*). As described earlier, both *mhf1Δ* and *mhf2Δ* mutants exhibit poor growth, and our data here show that this is not worsened when they are combined together or with *fml1Δ*. The poor growth hampers the comparison of genotoxin sensitivities, but nevertheless it is clear that both *mhf1Δ* and *mhf2Δ* exhibit similar levels of hypersensitivity to MMS and cisplatin, which is not further enhanced when combined with *fml1Δ*. This epistatic relationship indicates that MHF and Fml1 function in the same pathway for the repair/tolerance of ICLs and MMS-induced damage.

RETRACTED

**Figure 3.** MHF functions with Fml1 in the same DNA damage tolerance/repair pathway. (*a*) Spot assays comparing the growth and genotoxin sensitivities after 5 days of growth at 30°C for (*a*) strains MCW1221, MCW2080, MCW4639, MCW4777, MCW5127, MCW5790 and MCW5126, and (*b*) strains MCW1221, MCW2080, MCW5895 and MCW4405.

To see how important the interaction between Fml1 and MHF is for their ability to promote DNA repair, we compared the MMS and cisplatin sensitivities of a *fml1Δ* strain with one in which Y672, R674 and R678 in *fml1* were mutated to alanine and a *natMX4* marker inserted adjacent to its 3′ untranslated region (*fml1^AAA^::natMX4*; figure 3*b*). Interestingly, the *fml1^AAA^* mutant, although hypersensitive to MMS and cisplatin, is not as sensitive as a *fml1Δ* mutant. However, it exhibits the same sensitivity as a strain containing a truncated form of Fml1, in which the entire C-terminal domain from amino acid 604–834 is deleted (*fml1ΔC^1–603^*). Importantly, the hypersensitivity of both *fml1^AAA^* and *fml1ΔC^1–603^* mutants is not due to an altered level of Fml1 protein (see electronic supplementary material, figure S3) nor to the presence of the linked *natMX4* marker in these strains [12]. Together these data indicate that the critical role of Fml1's C-terminal domain is to mediate the interaction with MHF, and that without this Fml1 is still able to promote DNA repair, albeit at a reduced efficiency.

### 3.5. MHF functions with Fml1 to promote non-crossover recombination

Fml1 plays a major role in promoting NCO recombination both in mitotic and meiotic cells, and at least in the latter case MHF is also involved [19]. To further investigate the involvement of MHF in promoting NCO recombination, we used a plasmid gap repair assay, in which a plasmid containing a double-stranded gap within a copy of *ade6* is repaired by HR with a mutant copy (*ade6-M26*) on chromosome III, resulting in integration of the plasmid into the chromosome (CO) or recircularization of the plasmid (NCO) (figure 4*a*) [14]. In a wild-type strain, approximately 75% of the repaired plasmids contain a fully restored copy of *ade6^+^* resulting from a gene conversion (GC) event and only 10% of these are COs (figure 4*b*; electronic supplementary material, figure S4). A comparison of *fml1Δ*, *mhf1Δ* and *mhf2Δ* single and double mutants showed that they all exhibit wild-type levels of GC and gap repair, but, unlike wild-type, approximately 35% of *ade^+^* recombinants are COs (figure 4*b*; electronic supplementary material, figure S4). The similarity in the percentage of COs in both single and double mutant strains indicates that MHF plays an essential role in the Fml1-dependent pathway of NCO recombination in mitotic cells. Interestingly, the *fml1^AAA^* mutant exhibits only approximately 20% COs among *ade^+^* recombinants (figure 4*b*), which suggests that MHF may not need to interact with Fml1 in order to provide at least some assistance in promoting NCO recombination in mitotic cells.

RETRACTED

**Figure 4.** MHF promotes NCO recombination in both mitotic and meiotic cells. (*a*) Schematic of the plasmid gap repair assay. The filled circle indicates the position of the *M26* mutation. (*b*) Percentage of Ade^+^ transformants that are COs in strains MCW1193, MCW2096, MCW5345, MCW5346, MCW5790, MCW5983, MCW4893 and MCW6001. Values are means from three experiments ±s.d. (*c*) Schematic of the meiotic recombination assay showing the different types of CO and NCO recombinants that can be associated with an *ade6^+^* convertant. The filled circles indicate the position of the *3083* and *L469* mutations. (*d*) Percentage of CO associated with GC events at *ade6-3083* from wild-type and mutant crosses (see electronic supplementary material, table S1). Values are means from at least six crosses ±s.d. Statistical significance in comparison with wild-type and *fml1^+^::natMX4* is *p < 0.01.

MHF supports Fml1 in directing NCO recombination during meiosis [19]. To see whether the interaction between these proteins is important for this, we compared the percentage of COs associated with GC at the *ade6-3083* meiotic recombination hotspot in wild-type, *fml1Δ* and *fml1^AAA^* strains (figure 4*c*,*d*; electronic supplementary material, table S1). As seen previously, there is a small but significant increase in the percentage of COs associated with GC in a *fml1Δ* mutant compared with wild-type. A similar increase is also seen in the *fml1^AAA^* mutant, indicating that the interaction between Fml1 and MHF is important for directing NCO recombination during meiosis.

RETRACTED

### 3.6. MHF functions with Fml1 to promote gene conversion at blocked replication forks

Replication fork stalling at the *RTS1* protein–DNA barrier induces Rad51-dependent recombination, which can give rise to both GC (conversion-types) and deletions (deletion-types) between flanking *ade6^−^* heteroalleles (figure 5*a*) [30]. Fml1 plays a role here in promoting GC, probably by catalysing the reversal of the stalled fork, and recent work has implicated Mhf2 in assisting it in this function [12,14,22]. To confirm that MHF works with Fml1 in promoting GC at the *RTS1* barrier, we compared the frequency of *ade^+^* deletion- and conversion-types in *fml1Δ*, *mhf1Δ* and *mhf2Δ* single and double mutant strains, and in the *fml1^AAA^* mutant (figure 5*b*,*c*). Consistent with published data, absence of *fml1* has no effect on the frequency of deletion-types, but reduces conversion-types by approximately sevenfold. Both *mhf1Δ* and *mhf2Δ* single mutants likewise show a reduction (approx. threefold) in conversion-type frequency, but interestingly exhibit a small increase in deletion-types. Importantly, both *fml1Δ* *mhf1Δ* and *fml1Δ* *mhf2Δ* double mutants exhibit essentially the same deletion-type and conversion-type frequency as a *fml1Δ* single mutant. Similar to what was seen in the plasmid gap repair assay, the *fml1^AAA^* mutant exhibits a more modest effect on recombination than *fml1Δ*, with a reduction in conversion-types of twofold when compared with a *fml1^+^::natMX4* strain, which exhibits slightly higher recombinant frequencies than a wild-type without the *natMX4* marker. Altogether these data indicate that MHF promotes Fml1-dependent GC at stalled replication forks, and can do so at a reduced level even when unable to interact with Fml1's C-terminal domain. In the absence of MHF, Fml1 retains some ability to act but at a much reduced efficiency. Moreover, without MHF Fml1 may act in an aberrant fashion to promote the formation of deletion-types.

**Figure 5.** MHF functions with Fml1 to promote *RTS1*-induced direct repeat recombination. (*a*) Schematic of the recombination substrate on chromosome III, including the two classes of Ade^+^ recombinant product. (*b*) Deletion-type frequencies and (*c*) conversion-type frequencies in strains MCW4713, MCW3060, MCW4770, MCW5217, MCW5218, MCW5220, MCW4797 and MCW5932. All values are mean±s.d. Statistical significance in comparison with wild-type and *fml1^+^::natMX4* is *p < 0.01 and **p < 0.001.

### 3.7. MHF localizes to non-centromeric sites in a Fml1-dependent fashion

As shown in figure 1*b*, Mhf1-GFP co-localizes with the centromeric protein Mis6, consistent with it being a component of the CCAN. However, unlike Mis6, it also forms a speckling of fluorescence throughout the rest of the nucleus, which might represent its localization to sites across the genome where Fml1 is actively engaged in DNA repair and recombination. To investigate this, we assessed whether Mhf1-GFP localization is affected by deletion of *fml1* (figure 6; electronic supplementary material, figure S5). In a *fml1Δ* strain, Mhf1-GFP centromeric localization appears unaltered. By contrast, its wider distribution throughout the nucleus is lost or greatly diminished in almost all cells, and this is also true in a *fml1^AAA^* strain. This loss in general nuclear fluorescence is not due to a change in the amount of Mhf1-GFP, which is the same in both wild-type and *fml1* mutant strains (see electronic supplementary material, figure S6). To see whether the non-centromeric localization of MHF is dependent on Fml1's catalytic activity, we assessed Mhf1-GFP fluorescence in a *fml1^D196N^* strain, which contains a mutation in Fml1's helicase motif II that destroys its ATPase activity (and therefore its ability to unwind and branch migrate DNA junctions) without affecting its DNA binding [12]. Similar to the wild-type strain, Mhf1-GFP localized to both centromeric and non-centromeric sites throughout the nuclei of *fml1^D196N^* mutant cells (figure 6; electronic supplementary material, figure S5). Altogether these data indicate that MHF is recruited to and/or retained at non-centromeric chromosomal sites through its interaction with Fml1.

RETRACTED

**Figure 6.** Nuclear localization of Mhf1-GFP in wild-type and *fml1* mutant cells. The strains are MCW5846, MCW5963, MCW6152 and MCW6132.

### 3.8. Fml1 limits mitotic bridge and tail formation

In human cells, the FA pathway plays a role in limiting the occurrence of DNA bridges connecting segregating sister chromatids during mitosis [31]. To see whether Fml1 plays a similar role in *S. pombe*, we analysed binucleate cells from asynchronously growing cultures of wild-type and *fml1Δ* strains, using DAPI to stain the DNA (figure 7*a*,*b*). Only approximately 3% of wild-type binucleate cells exhibit a DNA bridge between the two masses of segregating DNA (figure 7*c*). By contrast, approximately 25% of *fml1Δ* binucleates exhibit a DNA bridge, albeit some of these are discontinuous and therefore perhaps better described as DNA tails with a small gap at or near the midpoint between the main DNA masses (figure 7*b*,*c*). The bridges and tails in the *fml1Δ* strain are also on average longer than those seen in wild-type cells (figure 7*d*). A similar frequency and length of bridges and tails was also seen among *fml1^D196N^* binucleates, whereas in a *fml1^AAA^* mutant their frequency is less, albeit still fivefold more than in a wild-type (figure 7*c*,*d*). Altogether these data indicate that Fml1's catalytic activity and interaction with MHF are needed for the efficient and timely resolution of DNA connections between sister chromatids.

RETRACTED

**Figure 7.** Mitotic DNA bridges in wild-type and *fml1* mutant cells. (*a*) Examples of wild-type cells undergoing mitosis. (*b*) Examples of *fml1Δ* mutant cells exhibiting a mitotic DNA bridge (top row) and tails (bottom row). (*c*) Frequency of mitotic DNA bridges/tails and (*d*) length of mitotic DNA bridges in strains MCW1221, MCW2080, MCW4778 and MCW5895. In all cases, values are mean±s.d. (*e*) Examples of Mhf1-GFP co-localizing with mitotic DNA bridges/tails in wild-type (MCW5846) and *fml1^D196N^* mutant cells (MCW6132).

### 3.9. MHF localizes to mitotic bridges and tails in a Fml1-dependent fashion

In human cells, immunostaining for FANCM has revealed that it forms bridges between segregating DNA in telophase, suggesting that it plays a role during this late stage of mitosis to resolve persistent connections between sister chromatids [31]. Similarly, Mhf1-GFP localizes to more than 90% of the mitotic DNA bridges or tails detected in wild-type cells by DAPI staining (figure 7*e*; electronic supplementary material, figure S7). This localization is far more striking in *fml1^D196N^* cells, which exhibit a greater frequency and length of bridges and tails than wild-type (figure 7*e*; electronic supplementary material, figure S7). In a few cases, we also observed Mhf1-GFP localizing to the region between the segregating DNA masses when no DNA bridge or tail was detected by DAPI staining (see electronic supplementary material, figure S7). Importantly, the localization of Mhf1-GFP to mitotic DNA bridges and tails is lost or greatly diminished in both *fml1Δ* and *fml1^AAA^* mutants (see electronic supplementary material, figure S7). Altogether these data indicate that MHF is recruited to and/or retained at mitotic DNA bridges and tails through its interaction with Fml1. The fact that these bridges are occasionally detected in wild-type cells suggests that Fml1 together with MHF can act as late as mitosis to resolve connections between sister chromatids.

### 3.10. Mus81–Eme1 functions as a failsafe for resolving sister chromatid connections in the absence of Fml1

Even though the frequency of mitotic DNA bridges and tails increases in a *fml1Δ* mutant, this does not lead to a correspondingly high frequency of aberrant chromosome segregation among cells that have laid down a division septum (figure 8*a*,*b*). This suggests that DNA bridges are resolved prior to cytokinesis. A prime candidate for resolving DNA junctions between sister chromatids is the Mus81–Eme1 endonuclease, whose orthologue in budding yeast is activated during G2 and M phase by CDK- and Polo-like kinase-dependent phosphorylation of Mms4 (the orthologue of Eme1) [32,33]. Consistent with Mus81–Eme1 playing an important role in resolving sister chromatid junctions, a high frequency (approx. 40%) of *mus81Δ* binucleate cells exhibit mitotic DNA bridges, tails and lagging chromosomes (see electronic supplementary material, figure S8). Moreover, unlike in a *fml1Δ* mutant, there is a similarly high number of septated cells with aberrant chromosomal segregation, including ‘cut’ (where DNA spans the division septum), missegregation and failed segregation phenotypes (figure 8*a*,*b*). A *mus81Δ* *fml1Δ* double mutant exhibits a marked reduction in growth and viability compared with either single mutant [14], and this correlates with a range of abnormal cell and nuclear morphologies, including many cells in which the DNA appears to be fragmented, possibly as a consequence of aberrant chromosome segregation or as part of an apoptotic response. Among septated cells, the frequency of aberrant chromosome segregation is much higher than in either single mutant, although it should be noted that the nuclear fragmentation, which is prevalent in the double mutant, complicates this analysis (figure 8*b*). Altogether these data indicate that Mus81–Eme1 is able to process the majority of DNA junctions that would normally be dealt with by Fml1.

RETRACTED

**Figure 8.** Partial suppression of aberrant chromosome segregation and genotoxin sensitivity in a *fml1Δ* *mus81Δ* double mutant by deleting *rad51*. (*a*) Examples of aberrant chromosome segregation in septated *mus81Δ* (MCW1779) and *mus81Δ* *fml1Δ* (MCW2428) mutant cells. Arrowheads indicate the division septum. (*b*) Frequency of aberrant chromosome segregation among septated cells in strains MCW1221, MCW2080, MCW1088, MCW1779, MCW2428 and MCW4490. Values are based on the analysis of approximately 300 septated cells from three independent asynchronously growing cultures. (*c*) Spot assay comparing the growth and genotoxin sensitivity of strains MCW3792, MCW1235, MCW2428 and MCW4490. Plates were photographed after 5 days growth at 30°C.

*In vitro* Mus81–Eme1 and Fml1 can process a similar spectrum of DNA junctions, including model replication forks and recombination intermediates such as D-loops and HJs [4,34]. The frequency of aberrant chromosome segregation in a *fml1Δ* *mus81Δ* double mutant is reduced almost twofold by deleting *rad51* (figure 8*b*), and *rad51* deletion also partially suppresses the hypersensitivity of a *fml1Δ* *mus81Δ* double mutant to ultraviolet (UV) light and MMS, which are agents that induce HR (figure 8*c*). These data suggest that much of the impaired chromosome segregation in a *fml1Δ* *mus81Δ* mutant is due to unresolved recombination intermediates that presumably impede sister chromatid separation. The fact that *rad51* deletion does not improve the growth and viability of a *fml1Δ* *mus81Δ* mutant more fully is probably due to Mus81 also having a role in a Rad51-independent DNA repair pathway [35].

RETRACTED

## 4. Discussion

Recent studies have established that vertebrate MHF functions as a component of the CCAN as well as an accessory factor for FANCM; however, it has been unclear whether these functions are entirely distinct or overlap. In HeLa cells, transiently transfected GFP-FANCM localizes to centromeres in an MHF1-dependent fashion, suggesting that it plays a role there in humans [23]. However, we have shown that, at least in fission yeast, MHF's function at the centromere is distinct from its role in supporting Fml1 in DNA repair and recombination. This conclusion is based on our observations that Mhf1-GFP localizes to centromeres in a Fml1-independent manner, and that, unlike a *fml1Δ* mutant, *mhf1/2Δ* mutants exhibit poor viability and high rates of meiotic chromosome missegregation. Although these data do not exclude the possibility that Fml1 functions at centromeres together with MHF, they do indicate that any role it might play there is non-essential.

Similar to human MHF, fission yeast MHF binds linear dsDNA but not ssDNA (see electronic supplementary material, figure S2; S.B. & M.C.W. 2013, unpublished data), whereas the helicase domains of both FANCM and Fml1 bind ssDNA and branched dsDNA structures but not linear dsDNA [4,22]. The Fml1–MHF complex is therefore endowed with the ability to bind all of the constituent parts of a stalled replication fork or D-loop, forming multiple protein–DNA contacts that presumably enable efficient targeting of these substrates *in vivo*. Moreover, the interaction between MHF and FANCM/Fml1 appears to generate an additional DNA binding site, which further enhances this ability of the complex [23] (figure 2*i*). Unsurprisingly, MHF is needed for the localization of FANCM to chromatin and its efficient recruitment to DNA ICLs [22,23]. Our data indicate that this dependency is likely to be reciprocal as Mhf1-GFP exhibits reduced or no localization to non-centromeric chromatin when unable to interact with Fml1 (because Fml1 is either deleted or mutated in its MHF interaction domain). Interdependence between both components of the FANCM/Fml1–MHF complex for localizing to non-centromeric chromatin would accord with its synergistic increase in DNA binding *in vitro* [22,23].

RETRACTED

MHF supports Fml1 in promoting NCO meiotic recombination and Rad51-dependent recombination at blocked replication forks [19,22]. We have shown here that it is also essential for Fml1's role in CO avoidance during mitotic DSB repair, and works together with Fml1 in promoting the tolerance/repair of both MMS and cisplatin-induced DNA damage. However, at least for promoting *RTS1*-induced direct repeat recombination, it is evident that Fml1 retains some ability to act without MHF. This is also true in chicken DT40 cells where deletion of FANCM results in a bigger increase in SCE than deletion of MHF1 [22]. More surprisingly, the interaction between Fml1 and MHF, at least mediated by Fml1's C-terminal domain, is not essential for MHF to make a contribution to Fml1-mediated DNA repair and recombination. Of course, we cannot be certain that the Y672A, R674A and R678A mutations generated in our study totally prevent Fml1 from interacting with MHF *in vivo*, which could occur additionally via unknown intermediary proteins and/or as a consequence of post-translational modification.

Replication forks blocked at *RTS1* are restarted by a recombination-dependent process [36], and therefore the reduction in *RTS1*-induced GC in both *fml1Δ* and *mhf1/2Δ* mutants probably reflects the fact that Fml1–MHF is a key component of the replication restart machinery. Indeed FANCM's ATPase activity has been shown to be important for stabilizing and restarting stalled replication forks in human cells [37]. Fml1's ability to catalyse fork reversal, which is probably enhanced by MHF, would generate a substrate for the recruitment of other recombination proteins, leading ultimately to the assembly of a Rad51-DNA filament, which catalyses the key step of strand invasion that reprimes DNA synthesis [12,14]. Without a fully functional Fml1–MHF complex replication restart would be impaired, and this could result in unreplicated regions of the genome persisting into mitosis, leading to an increase in mitotic DNA bridges (as observed in *fml1Δ*, *fml1^D196N^* and *fml1^AAA^* mutants). A similar scenario has been proposed to explain the increase in ultrafine anaphase bridges (UFBs) detected by immunostaining for the BLM DNA helicase in FANCM-depleted cells [31]. However, a failure to resolve recombination intermediates (i.e. D-loops and HJs) between sister chromatids could also account for the occurrence of mitotic DNA bridges in the *fml1* mutants. The possibility that some UFBs in human cells are caused by unresolved recombination intermediates has been largely discounted because UFB occurrence increases upon deletion of RAD51 [38]. However, in *S. pombe*, deletion of Rad51 and its key mediator Rad52, which together are responsible for all recombination-dependent replication restart (RDR) [36], results in a relatively small increase in the frequency of mitotic DNA bridges compared with a *fml1Δ* mutant (L.F. & M.C.W. 2013, unpublished data). Therefore, a failure to promote RDR cannot account for all of the mitotic DNA bridges that are observed when Fml1 is absent or impaired.

RETRACTED

A failure of FANCM to prevent/resolve UFBs correlates with an increase in multinucleated cells, which are thought to arise as a consequence of cytokinesis failure due to DNA being trapped in the cleavage furrow [31]. In *S. pombe*, septation proceeds even when DNA spans the division plane, resulting in cut phenotypes and uneven distribution of DNA between daughter cells [39,40]. Interestingly, very few of the mitotic DNA bridges in a *fml1Δ* mutant give rise to a cut or chromosome missegregation phenotype, indicating that alternative pathways of restarting stalled replication forks and processing recombination intermediates are able to act during mitosis to achieve sister chromatid separation prior to septation. At least one of these pathways appears to depend on Mus81–Eme1 since a *mus81Δ* *fml1Δ* double mutant exhibits a synergistic increase in chromosome missegregation and cell inviability. Importantly, these phenotypes are partially suppressed by deleting *rad51*, suggesting that some of the aberrant chromosome segregation is due to unresolved recombination intermediates. Mus81–Eme1's ability to act late in the cell cycle to resolve recombination intermediates accords with the finding in budding yeast that Mus81–Mms4 nucleolytic activity is activated in G2 and M phase [32,33]. Intriguingly, while Mus81–Eme1 appears to be able to resolve most of the recombination intermediates that accumulate in a *fml1Δ* mutant, the reverse is not true, as the majority of mitotic DNA bridges in a *mus81Δ* mutant seemingly give rise to cut and chromosome missegregation phenotypes. Single HJs formed during the repair of broken replication forks may account for these bridges, as neither Fml1 nor RecQ helicase-dependent double HJ dissolution would be able to substitute effectively for Mus81–Eme1 in resolving them productively [34].

One of the intriguing observations in our study is the speckled localization of Mhf1-GFP at non-centromeric sites throughout the nucleus, which depends on MHF's interaction with Fml1 but not on Fml1's ATPase activity. This pattern of localization is observed in essentially all cells within an asynchronously growing population, and presumably represents binding of Fml1–MHF or Fml1-dependent deposition of MHF to multiple genomic sites. Given MHF's potential to associate with other histone-fold proteins [22,25], it is possible that it forms distinct regions of chromatin at sites where replication forks have been perturbed or recombination enacted. Such chromatin could persist until its displacement in the following S-phase. Enrichment of Mhf1-GFP on mitotic DNA bridges may therefore represent either the redeployment of Fml1–MHF to replication/recombination intermediates in M-phase or its retention at these sites following earlier recruitment in S- or G2-phase. The former is certainly possible because in human cells FANCM has been shown to localize to UFBs in telophase [31]. Regardless of when it is recruited, Mhf1-GFP's presence on bridges suggests that Fml1–MHF is able to act during the late stages of the cell cycle to promote sister chromatid segregation.

RETRACTED

MHF is a member of a growing list of CCAN proteins that also function in DNA repair/recombination [41]. It has been speculated that recombination might play a role in proper centromere function [42], and if true this would provide a link between these seemingly disparate processes. However, at least in the case of MHF, its recombination function, which is rooted in its interaction with Fml1, is distinct from its key centromeric role. Nevertheless, it is intriguing to note that both its functions share a common aim in promoting chromosome segregation. Defining the evolutionary origin of this dual role presents an interesting challenge for future research.

## 5. Material and methods

### 5.1. *Schizosaccharomyces pombe* strains and plasmids

*Schizosaccharomyces pombe* strains are listed in electronic supplementary material, table S2. The *mhf1Δ*::*kanMX6* and *mhf2Δ*::*natMX4* strains were made by gene targeting using derivatives of pFA6a-kanMX6 [43] (pMW871) and pAG25 [44] (pMW872), respectively. The initial gene deletion was made in a diploid *S. pombe* strain from which haploid segregants were obtained. The *mhf1*::*GFP*-*kanMX6* strain was made by gene targeting directly in a haploid *S. pombe* strain using a derivative of pFA6a-GFP(S65 T)-kanMX6 [43] (pCB1). Similarly, *fml1^AAA^*::*natMX4*, *fml1ΔC^1–603^*::*natMX4, fml1^+^*::*13Myc*-*natMX4*, *fml1^AAA^*::*13Myc*-*natMX4* and *fml1ΔC^1–603^*::*13Myc*-*natMX4* strains were made by gene targeting in a haploid *S. pombe* strain using derivatives of pAG25 (pJBB79, pJBB9, pJBB28, pJBB81 and pJBB7, respectively). The plasmids for expressing full-length or fragments of Fml1 fused to MBP are all derivatives of pMAL-c2x (New England BioLabs) with a *Bam*HI–*Xba*I insert encoding the stated portion of Fml1. The plasmid for co-expressing Mhf1 and His-tagged Mhf2 (pMW891) was made by first cloning the cDNA for *mhf2* as an *Nde*I–*Bam*HI fragment into pET14b to make pMW884. A *Bgl*II–*Sal*I fragment containing the T7 promoter and *mhf1* cDNA from the pT7-7 derivative pMW889 was then cloned into these sites in pMW884. The plasmid for co-expressing Mhf1, His-tagged Mhf2 and Fml1^576–725^ (pCB6) was made by amplifying the T7 promoter and *fml1^576–725^* fragment from the pT7-7 derivative pCB5 and cloning this as a *Nhe*I fragment into pMW891. All plasmids were verified by DNA sequencing.

RETRACTED

### 5.2. Media and genetic methods

Media and genetic methods followed standard protocols [45]. The complete and minimal media were yeast extract with supplements (YES) and Edinburgh minimal medium plus 3.7 mg ml^−1^ sodium glutamate (EMMG), plus appropriate amino acids (0.25 mg ml^−1^), respectively. Sporulation of crosses was performed on malt extract agar (MEA). Low adenine media (YELA) was supplemented with 0.01 mg ml^−1^ adenine. Ade^+^ recombinants were selected on YES lacking adenine and supplemented with 0.2 mg ml^−1^ guanine to prevent uptake of residual adenine.

### 5.3. Spot assays

Exponentially growing cells from liquid cultures were harvested, washed and resuspended in water at a density of 1×10^7^–1×10^3^ cellsml^−1^. Aliquots (10 µl) of the cell suspensions were spotted onto YES agar plates containing genotoxins as indicated. For UV, plates were irradiated using a Stratalinker (Stratagene). Plates were photographed after 3–5 days growth at 30°C as indicated.

### 5.4. Microscopy

Cells from an exponentially growing culture in YES were harvested and fixed with 70% ethanol for subsequent microscopy. The fixed cells were stained with DAPI and analysed using an Olympus BX50 epifluorescence microscope equipped with the appropriate filter sets to detect blue, green and red fluorescence (Chroma Technology, VT). Black and white images were acquired with a CoolSNAP HQ^2^ CCD camera (Photometrics, AZ) controlled by MetaMorph software (v. 7.7.3.0, Molecular Devices, CA). Images were pseudo-coloured and overlayed using Photoshop CS5 (v. 12.0, Adobe Systems, CA).

### 5.5. Recombination assays

The direct repeat recombination, plasmid gap repair and meiotic recombination assays have been described previously [14,30,46,47]. Two sample *t*-tests were used to determine the statistical significance of differences in recombination values between strains unless otherwise stated.

### 5.6. Protein expression and purification

A 1 l culture of *E. coli* BL21 (DE3) CodonPlus-RIL cells (Stratagene) transformed with pMW891 was grown with aeration at 25°C in LB broth containing 50 μg ml^–1^ ampicillin and 20 μg ml^−1^ chloramphenicol to an A_600_ of 0.5. Mhf1-HisMhf2 was induced by adding IPTG to a final concentration of 0.5 mM, following which the cells were grown with aeration at 25°C for a further 5 h. The cells were then harvested by centrifugation, resuspended in 20 ml Buffer H (50 mM potassium phosphate, pH 8.0, 0.3 M NaCl, 10% glycerol) and frozen at −80°C until needed. The frozen cells were defrosted and mixed with 1% Triton X-100, 10 mM β-mercaptoethanol and EDTA-free protease inhibitor cocktail (Roche) before passage through a French pressure cell at 19 000 p.s.i. All subsequent steps were performed at 4°C. The lysates were cleared by centrifugation at 19 000*g* for 50 min, and the supernatant was loaded directly onto a 1 ml nickel-nitrilotriacetic acid Superflow column (Qiagen) that had been pre-equilibrated with Buffer H. The column was then washed with 60 ml of Buffer H plus 20 mM imidazole before eluting bound Mhf1-HisMhf2 with Buffer H plus 100 mM imidazole into three 1 ml fractions. The second 1 ml fraction contained the peak of Mhf1-HisMhf2 and was loaded directly onto a HiLoad 16/60 Superdex 200 gel filtration column (Amersham Biosciences), which was then developed with 120 ml of Buffer A (50 mM Tris–HCl, pH8.0, 1 mM EDTA, 1 mM DTT, 10% glycerol) plus 0.3 M NaCl. Fractions of 2 ml were collected, and the peak fractions containing Mhf1-HisMhf2 (fractions 36–42) were pooled, diluted with an equal volume of Buffer A and loaded onto a 1 ml Hi-Trap Heparin column (GE Healthcare). The column was then washed with 5 ml of Buffer A plus 0.1 M NaCl before eluting bound protein with an 18 ml linear gradient from 0.1 to 1.0 M NaCl. The peak of Mhf1-HisMhf2 eluted between 0.41 and 0.43 M NaCl, and these fractions were pooled and stored as aliquots at −80°C.

RETRACTED

The purification of Fml1^576–725^-Mhf1-HisMhf2 followed the same protocol as for Mhf1-HisMhf2 except the expression plasmid was pCB6 and the final heparin step was omitted. The peak of Fml1^576–725^-Mhf1-HisMhf2 eluted from the gel filtration column in fractions 34–36, and these fractions were pooled and stored as aliquots at −80°C.

Both full-length Fml1 and fragments of it were expressed as fusion proteins with MBP from the appropriate pMAL-c2x derivative in BL21 (DE3) CodonPlus-RIL cells. Cells were grown as 100 ml cultures at 25°C with aeration in LB broth containing 50 μg ml^−1^ ampicillin and 20 μg ml^−1^ chloramphenicol. At a cell density corresponding to an A_600_ of 0.6, IPTG was added to a final concentration of 250 μM and incubation continued for a further 12 h at 18°C. Cells were then harvested by centrifugation and resuspended in 10 ml of Buffer M (20 mM Tris–HCl, pH 7.4, 200 mM NaCl, 1 mM EDTA, 10% glycerol). DTT (1 mM), Triton X-100 (1%) and PMSF (4 mM) were added to the sample before it was lysed by passage through a French pressure cell at 19 000 p.s.i. All subsequent steps were performed at 4°C. Cell debris was removed by centrifugation at 19 000*g* and the cleared lysate was then loaded onto a 0.5 ml amylose column (New England Biolabs) pre-equilibrated with Buffer M, which was then washed with 12 ml of Buffer M before eluting bound protein with Buffer M plus 10 mM maltose. Protein samples were pooled and stored as aliquots at −80°C.

In all cases, protein amounts were estimated using a Bio-Rad protein assay kit with bovine serum albumin as the standard.

### 5.7. Protein–protein interaction assay

Full-length Fml1 and fragments of Fml1 fused to MBP were immobilized on 100 μl amylose resin by incubating them for 2 h at 4°C on a rotating wheel. After removing unbound protein by washing with Buffer M, purified Mhf1-HisMhf2 was added and the mixture incubated for 3 h at 4°C on a rotating wheel. Unbound protein was removed by three consecutive 20 min washes with 0.5 ml Buffer M before eluting bound protein with Buffer M plus 10 mM maltose. Samples were then analysed for the presence of Mhf1-HisMhf2 by Western blotting using anti-polyhistidine antibody (Sigma).

### 5.8. DNA substrates

The ^32^P-labelled linear dsDNA substrate was made by annealing oligonucleotides 2 and 44 (5′-CAACGTCATAGACGATTACATTGCTAGGACATCTTTGCCCACGTTGACCC-3′) as described by Whitby & Dixon [48].

### 5.9. DNA binding assays

Reaction mixtures (20 µl) contained 1.1 nM ^32^P-labelled linear duplex DNA in buffer (25 mM Tris–HCl, pH 8.0, 1 mM DTT, 100 µg ml^−1^ bovine serum albumin, 6% glycerol) plus protein as indicated. Reactions were incubated on ice for 15 min and then loaded onto a 4% native polyacrylamide gel in low-ionic-strength buffer (6.7 mM Tris–HCl, pH 8.0, 3.3 mM sodium acetate, 2 mM EDTA) that had been pre-cooled at 4°C. Gels were run for 1 h and 45 min at 160 V with continuous buffer recirculation. Gels were then dried on 3 MM Whatman paper and analysed by Phosphor Imaging using a Fuji FLA3000 and Image Gauge software.

## Supplementary Material

Bhattacharjee et al Supplementary Material
